RETRACTED

# Mathematical modeling and numerical simulation of supercritical processing of drug nanoparticles optimization for green processing: AI analysis

**DOI:** 10.1371/journal.pone.0309242

**Published:** 2024-09-04

**Authors:** Khalid Aljohani

**Affiliations:** Department of Mechanical Engineering, College of Engineering in Al-Kharj, Prince Sattam Bin Abdulaziz University, Al-Kharj, Saudi Arabia; University of Oklahoma, UNITED STATES OF AMERICA

## Abstract

In recent decades, unfavorable solubility of novel therapeutic agents is considered as an important challenge in pharmaceutical industry. Supercritical carbon dioxide (SCCO_2_) is known as a green, cost-effective, high-performance, and promising solvent to develop the low solubility of drugs with the aim of enhancing their therapeutic effects. The prominent objective of this study is to improve and modify disparate predictive models through artificial intelligence (AI) to estimate the optimized value of the Oxaprozin solubility in SCCO_2_ system. In this paper, three different models were selected to develop models on a solubility dataset. Pressure (bar) and temperature (K) are the two inputs for each vector, and each vector has one output (solubility). Selected models include NU-SVM, Linear-SVM, and Decision Tree (DT). Models were optimized through hyper-parameters and assessed applying standard metrics. Considering R-squared metric, NU-SVM, Linear-SVM, and DT have scores of 0.994, 0.854, and 0.950, respectively. Also, they have RMSE error rates of 3.0982E-05, 1.5024E-04, and 1.1680E-04, respectively. Based on the evaluations made, NU-SVM was considered as the most precise method, and optimal values can be summarized as (T = 336.05 K, P = 400.0 bar, solubility = 0.00127) employing this model. Fig 4

## 1. Introduction

Recent efforts have focused on developing novel strategies for the efficient transportation of pharmaceutically active compounds to enhance the therapeutic efficacy of drugs [1, 2]. Despite great importance, the emergence of some challenges about the solubility and diffusivity of novel therapeutic agents has restricted their wide applications [3, 4]. Very low solubility of new therapeutic entities is known as an important drawback, which must be addressed in pharmaceutical industry. One of the most promising methods to enhance the solubility of therapeutic drugs is the use of supercritical fluids (SCFs) [5–7].

SCFs have now been identified as a promising alternative to poisonous organic solvents. Indeed, extensive industrial-based application of SCFs is not only because of their environmentally-benign characteristics in disparate processes but also because of its cost-effective nature and low flammability [7–10]. This green technique possesses great potential of application in pharmacology to solve the serious disadvantages of traditional technologies like spray-drying [11, 12]. SCFs can be considered as an individual phase beyond critical conditions, which their physical properties such as density and viscosity can be conveniently altered by setting the temperature and pressure [13]. CO_2_ is most employed as a SCF in pharmacology, owing to its exceptional benefits, including negligible cohesive energy and low density [14–16].

RETRACTED

Recently, application of artificial intelligence (AI) technique has found its high place in many areas of chemical engineering including separation, chemical reaction, and pharmaceuticals to estimate the obtained data of experimental investigations [17–20]. Techniques of support vector machines, ensembles, and tree-based models are used to solve problems. Machine learning models may now be used to investigate a broad range of problems with several input variables and multiple output values. Using these models, associations between inputs and outputs can be found [21–23]. Models selected for this study are Decision Tree (DT), NU-SVM, and Linear-SVM.

A decision tree (DT) is a solution to overcome regression and classification problems efficiently. This model uses a tree-based (hierarchical) concept. Nodes in the tree are divided into two or more subsets by branches that branch out from a central, root node that includes all data (leaf nodes). One or multiple outputs are severed from the others at each branch node in a DT [24–27]. In this study, we used a tree-based technique called decision tree regression or regression tree, which allows for the determination of actual outcomes [26, 28, 29].

We also used two support vector machine models, namely Linear SVM and NU-SVM. The Linear SVM is a machine learning model that is widely used for regression and function estimation tasks. It leverages a set of linear characteristic functions to estimate and identify the optimal hyperplane that separates the data. This model is effective for linearly separable data and provides a straightforward approach to regression problems [30].

The NU-SVM model, on the other hand, is a variant of the standard SVM that introduces a parameter to control the number of support vectors and margin errors. This model is particularly useful for datasets where a non-linear relationship exists between the input variables and the output. It aims to find a balance between the complexity of the model and its ability to generalize to new data, thus avoiding overfitting [31].

In order to select models, we initially evaluated a substantial number of machine learning models through a preliminary assessment. The selection was made based on the models that exhibited minimal overfitting and satisfactory accuracy. The primary innovative aspect of this research is the focus on addressing the issue of overfitting during model selection and optimization, a factor that is often overlooked in most similar studies.

RETRACTED

## 2. Data set

The dataset that was used for this investigation was obtained from reference [32], and it only contains 32 data vectors. Each vector consists of one output (solubility) and two input parameters, temperature and pressure. Table 1 provides an illustration of the dataset.

**Table 1:** The whole rows of the used dataset [32].

No.	Temperature (K)	Pressure (bar)	Solubility (mole fraction)
**1**	308	120	8.19E-05
**2**		160	1.58E-04
**3**		200	2.24E-04
**4**		240	2.80E-04
**5**		280	3.44E-04
**6**		320	4.06E-04
**7**		360	4.73E-04
**8**		400	5.33E-04
**9**	318	120	7.55E-05
**10**		160	1.41E-04
**11**		200	2.45E-04
**12**		240	3.56E-04
**13**		280	4.64E-04
**14**		320	5.58E-04
**15**		360	6.60E-04
**16**		400	7.66E-04
**17**	328	120	5.34E-05
**18**		160	1.28E-04
**19**		200	3.02E-04
**20**		240	4.14E-04
**21**		280	5.82E-04
**22**		320	7.87E-04
**23**		360	8.51E-04
**24**		400	1.03E-03
**25**	338	120	3.31E-05
**26**		160	9.09E-05
**27**		200	2.98E-04
**28**		240	4.81E-04
**29**		280	6.77E-04
**30**		320	8.89E-04
**31**		360	1.08E-03
**32**		400	1.24E-03

Fig 1 illustrates the Pearson plot of used dataset, which measures the strength and direction of the linear relationship between parameters such as temperature, pressure, and solubility of Oxaprozin in the SCCO_2_ system. The coefficient varies between -1 to 1, where 1 implies a perfect positive linear correlation, -1 shows a perfect negative linear correlation, and 0 shows no linear relationship. The plot’s color-coded matrix helps quickly identify strong correlations, providing insights into the data’s underlying patterns.

**Fig 1:** Pearson plot of solubility data.

## 3. Methodology

### 3.1 Linear SVM

The Support Vector Machine (SVM) is a widely used ML known for its effectiveness in regression and function estimation tasks, leveraging a set of linear characteristic functions. One of the primary kernels utilized in SVM is the linear kernel. It is employed to estimate and identify the optimal hyperplane that separates the data. This hyperplane, situated in n-dimensional space, is illustrated below [33, 34]:

$$w^{T}x+b=0$$

In the above equation, *w*^*T*^ illustrates the gradient vector and *x* illustrates the hyperplane point carrier. The data might then be linearly divided, with the y-intercept vector indicated by b and hard margin SVM used. In the support vector method, two parallel hyperplanes are employed in order to separate classes of samples. Soft margin SVM SSSVM was developed for situations in which data cannot be linearly separated. In [35], SVM regression method is developed, with the goal of allowing for some degree of tolerance in the SVM model [36, 37]:

$$min\;1/2w^{T}w\;S.t.\;|y_{i}-(w^{T}x_{i}+b)|<\epsilon$$

In which *y _i_*∈ *{−1,1}*.

RETRACTED

### 3.2 NU-SVM

The basic configuration of a set of data pair of values *{(x*_*1*_, *y*_*1*_*)*,…, *(x*_*n*_, *y*_*n*_*)}*. In Nu-SVM regression method, the goal is to find the non-linear relation depicted in the following function, as *f(x)* have to be near to *y*. Flatness is also a requirement which refers to the simplicity of the model. A flatter function means the model is less complex and is likely to generalize better to new, unseen data. This helps in avoiding overly complicated models that can fit noise in the training data.

Also, overfitting happens when a model learns the noise in the training step to the extent that it works poorly on new data. In NU-SVM, parameter C controls the balance between fitting the training data well and maintaining the model’s generalization ability. A higher C value can lead to overfitting, while a lower C value encourages a simpler, flatter model that is less likely to overfit. As a result of this study, we are looking for models that aren’t too over fitted [38, 39].


$$f(x)=w^{T}\Phi (x)+b$$

The non-linear mapping function *Փ(x)* is defined here as the bias. The feature space is transformed into a higher-dimensional space by *Փ(x)*. *w*^*T*^ is another name for the weights vector. Optimization is the primary objective of the problem. Ultimately, the aim of the challenge is to maximize the determined function’s closeness and flatness in order to ensure its success [40]:

$$\frac{1}{2}|\left\lceil w\right\rceil {|}^{2}+C\{Y.ɛ+\frac{1}{n}\sum_{i=1}^{n}\left(\xi +\xi^{*}\right)\}$$

Depending on the circumstances [40]:

$$y_{i}‐\langle w^{T}.Փ(x)\rangle -b\leq ɛ+\xi_{i}^{*},$$

$$\langle w^{T}.Փ(x)\rangle +b-y_{i}\leq ɛ+\xi_{i},$$

$$\xi_{i}^{*},\xi_{i}\geq 0$$

In the above equations, ɛ stands for a distance of *f(x)* from corresponding observed amount, also *ξ*, *ξ*_*i*_ represent extra slack variables [41], which states that *ξ* above ɛ error are acceptable differences in value. For example, the regularization value, defined as C, shows the tradeoff between parameter *f*’s flatness and the hyper-parameter tolerance for error more than ɛ.

As a result, *Y* (between 0 and 1) reflects the maximum allowed value on the equation of marginal errors in training amounts and the minimum allowed value on the proportion of support vectors. Dual formulations are characterized by generating the Lagrange function (L) [40]:

$$L:\frac{1}{2}|\left\lceil w\right\rceil {|}^{2}+C\left\{Y.ɛ+\frac{1}{n}\sum_{i=1}^{n}\left(\xi^{*}+\xi \right)\right\}-\frac{1}{n}\sum_{i=1}^{n}\left(\eta \xi +{\eta^{*}\xi }^{*}\right)-\frac{1}{n}\sum_{i=1}^{n}\left(ɛ+\xi_{i}+y_{i-}w^{T}.Փ(x)-b\right)-\frac{1}{n}\sum_{i=1}^{n}\left(ɛ+\xi_{i}+y_{i}+w^{T}.Փ(x)+b\right)-\beta ɛ$$

Therefore, Lagrange multipliers are *η*, η^*^, *a*, a^*^, *β* and *a*^(*)^ *= a*.a^*^ [42]:

*W* = $\sum_{i=1}^{n}(a_{i}-a_{i}^{*}).\;Փ(x)$ and it leads to a pair of optimization tasks

Maximizes—$\frac{1}{2}\sum_{i=1}^{n}\left(a_{i}{-a}_{i}^{*}\right).(a_{j}a_{j}^{*}).k(x_{i}x_{j})+\sum_{i=1}^{n}y_{i}(a_{i}{-a}_{i}^{*});$

$$\sum_{i=1}^{n}\left(a_{i}{-a}_{i}^{*}\right)=0$$

$$CY\geq \sum_{i=1}^{n}\left(a_{i}{-a}_{i}^{*}\right)$$

$$a_{i}{,a}_{i}^{*}\epsilon \left[0,\frac{C}{n}\right]$$

Using *K(x*_*i*_,*x*_*j*_*)* as an example, we can see that *K(x*_*i*_,*x*_*j*_*) = Փ(x*_*i*_*)*^*T*^.*Փ (x*_*j*_*)* The Lagrange multipliers a and a* are obtained as a result of solving the previous equation. The predicted function (L) is as follows when weight W is interchanged in the equations above [38, 39]:

$$f(x)=b+\sum_{n=1}^{n}(a_{i}-a_{i}^{*}{).k(x}_{i},x)$$

RETRACTED

### 3.3 Decision tree

Recent years have seen a rise in the use of decision tree prediction models (DT) as a machine learning technique. This strategy is particularly useful in issues like the current one, which involve some category data. A decision tree includes numerous terminal (leaf) nodes and several internal nodes (decision nodes). Based on one or more input attributes, each internal node separates the data into two halves, and this process repeats sequentially through the subtrees to the terminal nodes. The final predicate value is contained in each terminal node (regression and classification) [24, 28, 43, 44]. Fig 2 depicts an overall decision tree structure.

**Fig 2:** Schematic of a DT with 4 internal and 5 terminal nodes.

## 4. Results and discussions

After selecting the best values of hyper-parameters and implementation of models, their accuracy was evaluated. MAPE and RMSE are two kinds of statistical errors which are utilized to optimize the efficiency of proposed procedures [45, 46]:

$$RMSE=\sqrt{\frac{\sum_{i=1}^{n}{\left(t_{i}-o_{i}\right)}^{2}}{n}}$$

$$MAPE=\frac{(\sum_{i=1}^{n}\left|\frac{t_{i}-o_{i}}{t_{i}}\right|)\times 100}{n}$$

R^2^ (or Coefficient of Determination) is a measure of how much variance there is in the data [46]:

$$R^{2}=\frac{{(n\sum t_{i}o_{i}-\sum t_{i}\sum o_{i})}^{2}}{\left(n\sum t_{i}^{2}-{\left(\sum t_{i}\right)}^{2})-(n\sum a_{i}^{2}-{\left(\sum a_{i}\right)}^{2}\right)}$$

*n* is the size of dataset, *t* denotes the experimental data (target), and *o* denotes the results.

RETRACTED

RMSE measures the square root of the average squared differences between estimated and actual values, penalizing larger errors more significantly. A lower RMSE indicates a better fit of the model. MAPE provides the average absolute percent error between estimated and reference values, offering an intuitive percentage measure of accuracy. Lower MAPE values signify better performance.

Figs 3 to 5 compare the predicted values of Oxaprozin solubility in supercritical carbon dioxide (SCCO_2_) system versus those data obtained from experimental research applying Nu-SVM, Linear-SVM and Decision Three models. The precision of total and absolute error in the difference between actual and estimated results is shown by the prediction calculated by MAPE and RMSE. Low RMSE and MAPE values indicate that the estimated-out puts are in good agreement with the experimental data. Big numbers also show that predictions differ greatly from the actual outcome. In these figures, the green line renders the expected (actual) data, and the red and blue points present the test and train data, respectively. Comparison of the presented values in Table 2 confirms the superiority of Nu-SVM model in precision and accuracy than other predictive models. The cross-validation values (3-fold method) also show robustness and generality of this model.

**Fig 3:** Predicted versus expected values for Oxaprozin solubility in the supercritical carbon dioxide (SCCO_2_) system using the Nu-SVM model, indicating significant agreement between predicted and expected values.

**Fig 4:** Predicted versus expected values for Oxaprozin solubility in the SCCO_2_ system using the Linear-SVM model, highlighting a moderate level of agreement between predicted and expected values.

**Fig 5:** Predicted versus expected values for Oxaprozin solubility in the SCCO_2_ system using the decision tree (DT) model, showing a reasonable agreement between predicted and expected values.

**Table 2:** Comparative performance metrics of NU-SVM, Linear-SVM, and decision tree models for predicting Oxaprozin solubility in supercritical carbon dioxide.

Models	RMSE	R^2^	Mean CV R^2^	Std Dev CV R^2^	MAPE
**Nu-SVM**	3.0982E-05	0.994	0.96320	0.019243	2.093E-01
**Linear-SVM**	1.5024E-04	0.854	0.84214	0.087513	1.036E+00
**Decision Tree**	1.1680E-04	0.950	0.92739	0.113306	3.143E-01

Fig 6A shows a 3D graphical representation based on the NU-SVM model, illustrating the combined effects of temperature and pressure on Oxaprozin solubility in an SCCO_2_ system. This figure helps visualize how these parameters interact to influence solubility, highlighting optimal conditions for maximum solubility.

RETRACTED

**Fig 6:** a. Input-Output projection (NU-SVM). b. Predicted Solubility based on Temperature. c. Predicted Solubility based on Pressure.

Fig 6B and 6C provide 2D projections for evaluating the individual impacts of temperature and pressure on Oxaprozin solubility. Fig 6B depicts solubility as a function of temperature, showing a non-linear relationship where solubility initially decreases with increasing temperature before rising again. Fig 6C shows solubility as a function of pressure, demonstrating a more straightforward increase in solubility with higher pressure, due to enhanced solvent density. These figures collectively offer a detailed view of how temperature and pressure affect Oxaprozin solubility in an SCCO_2_ system, emphasizing the importance of optimizing both parameters to enhance drug solubility.

As shown, increasing the pressure has a positive effect on the solubility of Oxaprozin in the SCCO_2_ fluid system. Better speaking, pressure can be considered as a driving force for the density of SCFs and increase its value by enhancing the molecular compaction. The increase in density enhances the solvating power of SCCO_2_ and therefore the solubility of medicine. Against straightforward impact of pressure on increasing the solubility of medicine in SCCO_2_ fluid system, Temperature has a more complicated impact. It is important to note that by increasing the temperature, the value of solvent’s pressure sublimation increases, while the amount of solvent’s density significantly reduces. Increase in the sublimation pressure enhances the Oxaprozin solubility in SCCO_2_ fluid system but decrease in the density of solvent deteriorates the solubility. Whenever the pressure of the SCCO_2_ fluid system goes beyond the cross-over pressure, the positive effect of sublimation pressure dominates the negative effect of solvent density reduction and thus, the solubility of Oxaprozin in SCF increases. Whenever the pressure of the SCCO_2_ fluid system is below the cross-over pressure, the negative impact of density reduction overcomes the positive influence of the increment of the solvent’s pressure sublimation and therefore, enhances the Oxaprozin solubility in SCCO_2_ fluid system. According to Table 3, 336.05 K and 400 bar are the optimized values of the pressure and the temperature for achieving the maximum Oxaprozin solubility. The first row in this table represents the most favorable data point, while the other rows contain projections for alternative data points.

**Table 3:** Optimal temperature and pressure values for maximum Oxaprozin solubility in supercritical carbon dioxide (SCCO_2_) system alongside with predictions for some other random data points.

Temperature (K)	Pressure (bar)	Solubility
336.05	400.0	0.00127
318.0	200.0	0.000249
328.0	160.0	0.000107
338.0	400.0	0.001180
308.0	320.0	0.000404

RETRACTED

## 5. Conclusion

In this paper, the optimized value of Oxaprozin solubility in SCCO_2_ system in different ranges of temperature and pressure has been achieved via developing three predictive mathematical models based on ML and AI techniques. A solubility dataset with 32 data vectors was used in this study, and three different models were used to create models. Temperature and Pressure are input attributes for each vector, and the single output is the result (solubility). Models that were selected include NU-SVM, Linear-SVM, and Decision Trees (DT). Hyper-parameter optimization and standard metrics employed for evaluation of the models. In the R-squared metric, NU-SVM (0.994), Linear-SVM (0.854), and DT (0.995) were obtained. In addition, they have RMSE error rates of 3.0982E-05, 1.5024E-04, and 1.1680E-04, respectively. To summarize, NU-SVM proved to be the most accurate model, with optimal values of (T = 336.05 K, P = 400.0 bar, 0.00127) obtained by using this model.

## References

[1] KankalaR.K., et al., Supercritical fluid technology: an emphasis on drug delivery and related biomedical applications. Advanced healthcare materials, 2017. 6(16): p. 1700433. doi: 10.1002/adhm.201700433 28752598 PMC5849475

[2] LangerR., New methods of drug delivery. Science, 1990. 249(4976): p. 1527–1533. doi: 10.1126/science.2218494 2218494

[3] DahanA. and MillerJ.M., The solubility–permeability interplay and its implications in formulation design and development for poorly soluble drugs. The AAPS journal, 2012. 14(2): p. 244–251. doi: 10.1208/s12248-012-9337-6 22391790 PMC3326160

[4] KhanK.U., et al., Overview of nanoparticulate strategies for solubility enhancement of poorly soluble drugs. Life Sciences, 2022: p. 120301. doi: 10.1016/j.lfs.2022.120301 34999114

[5] CarvalhoV.S., et al., Supercritical fluid adsorption of natural extracts: Technical, practical, and theoretical aspects. Journal of CO2 Utilization, 2022. 56: p. 101865.

[6] SodeifianG., et al., Measurement and modeling of metoclopramide hydrochloride (anti-emetic drug) solubility in supercritical carbon dioxide. Arabian Journal of Chemistry, 2022. 15(7): p. 103876.

[7] AbdelbassetW.K., et al., Development a novel robust method to enhance the solubility of Oxaprozin as nonsteroidal anti-inflammatory drug based on machine-learning. Scientific Reports, 2022. 12(1): p. 1–9.35908085 10.1038/s41598-022-17440-4PMC9338996

RETRACTED

[8] PasqualiI. and BettiniR., Are pharmaceutics really going supercritical? International journal of pharmaceutics, 2008. 364(2): p. 176–187. doi: 10.1016/j.ijpharm.2008.05.014 18597957

[9] GirotraP., SinghS.K., and NagpalK., Supercritical fluid technology: a promising approach in pharmaceutical research. Pharmaceutical development and technology, 2013. 18(1): p. 22–38. doi: 10.3109/10837450.2012.726998 23036159

[10] SekhonB.S., Supercritical fluid technology: an overview of pharmaceutical applications. International Journal of PharmTech Research, 2010. 2(1): p. 810–826.

[11] ZhanS., et al., Preparation of 5-Fu-loaded PLLA microparticles by supercritical fluid technology. Industrial & Engineering Chemistry Research, 2013. 52(8): p. 2852–2857.

[12] KompellaU.B. and KoushikK., Preparation of drug delivery systems using supercritical fluid technology. Critical Reviews™ in Therapeutic Drug Carrier Systems, 2001. 18(2). 11325031

[13] DaviesO.R., et al., Applications of supercritical CO2 in the fabrication of polymer systems for drug delivery and tissue engineering. Advanced drug delivery reviews, 2008. 60(3): p. 373–387. doi: 10.1016/j.addr.2006.12.001 18069079

[14] BaldinoL., ScognamiglioM., and ReverchonE., Supercritical fluid technologies applied to the extraction of compounds of industrial interest from Cannabis sativa L. and to their pharmaceutical formulations: A review. The Journal of Supercritical Fluids, 2020. 165: p. 104960.

[15] FrancoP. and De MarcoI., Nanoparticles and nanocrystals by supercritical CO2-assisted techniques for pharmaceutical applications: A review. Applied Sciences, 2021. 11(4): p. 1476.

[16] BaldinoL., ScognamiglioM., and ReverchonE., Supercritical CO2 elimination of solvent residues from active pharmaceutical ingredients: Beclometasone dipropionate and Budesonide. The Journal of Supercritical Fluids, 2021. 177: p. 105325.

[17] ApriyandiA., Application Of The Western Art Form Based On Artificial Intelligence. Acta Informatica Malaysia (AIM), 2020. 4(2): p. 45–46.

[18] MohagheghS.D., Recent developments in application of artificial intelligence in petroleum engineering. Journal of Petroleum Technology, 2005. 57(04): p. 86–91.

[19] SyahR., et al., Artificial Intelligence simulation of water treatment using nanostructure composite ordered materials. Journal of Molecular Liquids, 2022. 345: p. 117046.

[20] MittalS., et al., Artificial Intelligence based modeling of pervaporation process for alcohol dehydration. Materials Today: Proceedings, 2022. 50: p. 150–154.

[21] BishopC.M., Pattern recognition. Machine learning, 2006. 128(9).

[22] Rodriguez-GalianoV., et al., Machine learning predictive models for mineral prospectivity: An evaluation of neural networks, random forest, regression trees and support vector machines. Ore Geology Reviews, 2015. 71: p. 804–818.

RETRACTED

[23] GoodfellowI., BengioY., and CourvilleA., Machine learning basics. Deep learning, 2016. 1(7): p. 98–164.

[24] XuM., et al., Decision tree regression for soft classification of remote sensing data. Remote Sensing of Environment, 2005. 97(3): p. 322–336.

[25] BreimanL., et al., Classification and regression trees. 2017: Routledge.

[26] SafavianS.R. and LandgrebeD., A survey of decision tree classifier methodology. IEEE transactions on systems, man, and cybernetics, 1991. 21(3): p. 660–674.

[27] LiuY., et al., Computational simulation of mass transfer in membranes using hybrid machine learning models and computational fluid dynamics. Case Studies in Thermal Engineering, 2023. 47: p. 103086.

[28] MathuriaM., Decision tree analysis on j48 algorithm for data mining. Intrenational Journal of Advanced Research in Computer Science and Software Engineering, 2013. 3(6).

[29] RokachL. and MaimonO.Z., Data mining with decision trees: theory and applications. Vol. 69. 2007: World scientific.

[30] ZhangF. and O’DonnellL.J., Support vector regression, in Machine learning. 2020, Elsevier. p. 123–140.

[31] ChangC.-C. and LinC.-J., Training v-support vector regression: theory and algorithms. Neural computation, 2002. 14(8): p. 1959–1977.12180409 10.1162/089976602760128081

[32] KhoshmaramA., et al., Supercritical process for preparation of nanomedicine: Oxaprozin case study. Chemical Engineering & Technology, 2021. 44(2): p. 208–212.

[33] MangasarianO.L. and MusicantD.R., Robust linear and support vector regression. IEEE Transactions on Pattern Analysis and Machine Intelligence, 2000. 22(9): p. 950–955.

[34] MartinM. On-line support vector machine regression. in European Conference on Machine Learning. 2002. Springer.

[35] DruckerH., et al., Support vector regression machines. Advances in neural information processing systems, 1997. 9: p. 155–161.

[36] MoosaeiH., et al., Generalized twin support vector machines. Neural Processing Letters, 2021. 53(2): p. 1545–1564.

[37] SmolaA.J. and SchölkopfB., A tutorial on support vector regression. Statistics and computing, 2004. 14(3): p. 199–222.

[38] BurgesC.J., A tutorial on support vector machines for pattern recognition. Data mining and knowledge discovery, 1998. 2(2): p. 121–167.

[39] MeyerD., LeischF., and HornikK., The support vector machine under test. Neurocomputing, 2003. 55(1–2): p. 169–186.

[40] LafdaniE.K., NiaA.M., and AhmadiA., Daily suspended sediment load prediction using artificial neural networks and support vector machines. Journal of Hydrology, 2013. 478: p. 50–62.

RETRACTED

[41] CortesC. and VapnikV., Support-vector networks. Machine learning, 1995. 20(3): p. 273–297.

[42] LinJ.-Y., ChengC.-T., and ChauK.-W., Using support vector machines for long-term discharge prediction. Hydrological sciences journal, 2006. 51(4): p. 599–612.

[43] SongY.-Y. and YingL., Decision tree methods: applications for classification and prediction. Shanghai archives of psychiatry, 2015. 27(2): p. 130.10.11919/j.issn.1002-0829.215044PMC446685626120265

[44] YangL., et al., A regression tree approach using mathematical programming. Expert Systems with Applications, 2017. 78: p. 347–357.

[45] RahmanS.N.A., et al., The artificial neural network model (ANN) for Malaysian housing market analysis. Planning Malaysia, 2019. 17.

[46] BotchkarevA., Evaluating performance of regression machine learning models using multiple error metrics in azure machine learning studio. Available at SSRN 3177507, 2018.

